This article has been retracted.

# Keloid Core Factor CTRP3 Overexpression Significantly Controlled TGF-*β*1-Induced Propagation and Migration in Keloid Fibroblasts

**DOI:** 10.1155/2023/9638322

**Published:** 2023-04-12

**Authors:** Lin He, Chan Zhu, Huicong Dou, Xueyuan Yu, Jing Jia, Maoguo Shu

**Affiliations:** ^1^Department of Plastic, Aesthetic and Maxillofacial Surgery, The First Affiliated Hospital of Xi'an Jiaotong University, Xi'an 710061, China; ^2^Department of Burns and Cutaneous Surgery, Xijing Hospital, The Fourth Military Medical University, Xi'an 710032, China

## Abstract

**Purpose:**

Keloid is a type of benign fibrous proliferative tumor characterized by excessive scarring. C1q/TNF-related protein 3 (CTRP3) has been proven to possess antifibrotic effect. Here, we explored the role of CTRP3 in keloid. In the current research, we examined the influence of CTRP3 on keloid fibroblasts (KFs) and investigated the potential molecular mechanism.

**Methods:**

KF tissue specimens and adjacent normal fibroblast (NF) tissues were collected cultured from 10 keloid participants. For the TGF-*β*1 stimulation group, KFs were processed with human recombinant TGF-*β*1. Cell transfection of pcDNA3.1-CTRP3 or pcDNA3.1 was performed. The siRNA of CTRP3 (si-CTRP3) or negative control siRNA (si-scramble) was transfected into KFs.

**Results:**

CTRP3 was downregulated in keloid tissues and KFs. CTRP3 overexpression significantly controlled TGF-*β*1-induced propagation and migration in KFs. Col I, *α*-SMA, and fibronectin mRNA and protein levels were enhanced by TGF-*β*1 stimulation, whereas they were inhibited by CTRP3 overexpression. In contrast, CTRP3 knockdown exhibited the opposite effect. In addition, CTRP3 attenuated TGF-*β* receptors TRI and TRII in TGF-*β*1-induced KFs. Furthermore, CTRP3 prevented TGF-*β*1-stimulated nuclear translocation of smad2 and smad3 and suppressed the expression levels of p-smad2 and p-smad3 in KFs.

**Conclusion:**

CTRP3 exerted an antifibrotic role through inhibiting proliferation, migration, and ECM accumulation of KFs via regulating TGF-*β*1/Smad signal path.

## 1. Introduction

Keloid is a type of benign fibrous proliferative tumor spontaneously occurred in the skin or occurred following minor trauma or injury [1]. Keloid is characterized by excessive scarring and can occur on any part of the body such as shoulder, upper arm, anterior chest, and face [2]. In recent years, keloid has gained particular concern since it can cause aesthetically disfiguring and major functional impairment [3, 4]. Previous researches indicate that the formation/growth of keloid is clearly associated with various risk factors [5]. In order to develop more effective targets for the treatment of keloids in the future, further research focusing on changes in scar-related genes is needed [5].

C1q/TNF-related proteins (CTRPs) are a family of secreted proteins with specific structure [6]. CTRPs have attracted much interest because of its wide-ranging effects upon survival signaling, inflammation, metabolism, and insulin sensitizing [7]. Previous study has indicated that CTRPs may be involved in the pathogenesis of scar formation. CTRP6 was found to be downregulated in dermal fibroblasts in response to TGF-*β*1 and inhibit fibrogenesis in human dermal fibroblasts through regulating the cell propagation and Col I and *α*-SMA [8].

CTRP3 is a unique member of the CTRP family and circulates in the blood and exerts broad physiological functions [9]. For instance, CTRP3 increases liver lipid metabolism, improves heart attack, inhibits inflammation, prevents arthritis and repairs cartilage, and regulates bone cancers osteosarcoma and chondroblastoma [9]. Moreover, CTRP3 is emerging as molecule potentially involved in skin lesions in late-stage systemic sclerosis. Moreover, serum CTRP3 level may be used as predictive and diagnostic factor in systemic sclerosis [10]. This research was designed to test the influence of CTRP3 on KFs and the potential related signaling pathway.

## 2. Materials and Methods

### 2.1. Clinical Tissues

KF tissue specimens and adjacent normal fibroblast (NF) tissues were collected from 10 keloid participants. The patients received surgical procedures between July 2017 and December 2018 at The First Affiliated Hospital of Xi'an Jiaotong University (Xi'an, China). The procedures were approved by the Ethics Committee of our hospital (No. 2016-52/251). The patients were informed the purpose of the study, and all participants affixed the informed consent.

### 2.2. Cell Culturing

NFs and primary KFs were, respectively, isolated as described previously [11]. The obtained cells were resuspended in DMEM (Gibco, Grand Island, NY, the United States) with 10% FBS (Gibco). Fibroblasts at passages of 3 to 5 were applied in the further experiments. For the TGF-*β*1 stimulation group, KFs were processed with human recombinant TGF-*β*1 (5 ng/ml; Sigma, St. Louis, MO, the United States) for 24 h.

### 2.3. Cell Transfection

A CTRP3-overexpressing plasmid pcDNA3.1-CTRP3 was generated. Cell transfection of pcDNA3.1-CTRP3 or pcDNA3.1 was performed with Lipofectamine 3000 Reagent (Invitrogen, Carlsbad, CA, USA). The siRNA of CTRP3 (si-CTRP3) or negative control siRNA (si-scramble) (GenePharma, Shanghai, China) was transfected into KFs via Lipofectamine RNAiMAX Transfection Reagent (Invitrogen).

### 2.4. RT-qPCR

Total RNAs isolated from clinical samples and fibroblasts were applied to compound cDNA with a reverse transcriptase kit (Takara, Dalian, China). Then, the RT-PCR was performed in the standard way via SYBR Green Master Mix (Takara) with corresponding primers of CTRP3, type I collagen (Col I), fibronectin, *α*-smooth muscle actin (*α*-SMA), or *β*-actin.

### 2.5. WB

Total proteins of clinical samples and fibroblasts were subjected to WB analysis with specific first antibodies including anti-CTRP3, anti-Col I, anti-fibronectin, anti-*α*-SMA, anti-TGF-*β* RI, anti-TGF-*β* RII, anti-smad2, anti-p-smad2, anti-smad3, anti-p-smad3 (1 : 1000), and anti-*β*-actin (diluted in 1 : 1000-1 : 1500; Abcam or Santa Cruz Biotechnology), followed by HRP-conjugated second antibodies (diluted in 1 : 5000; Abcam). The protein bands were developed via an ECL reagent (Thermo Fisher Scientific, Waltham, MA, the United States).

### 2.6. Cell Proliferation Assay

Briefly, 20 *μ*l of MTT solution (5 mg/ml; Sigma) was supplemented to KFs and cultivated for 4 h. Afterwards, the medium was changed with 150 *μ*l of dimethyl sulfoxide (DMSO; Sigma) and gently shaken for 10 min. Finally, absorbance was monitored using a microplate reader.

### 2.7. Cell Migration Test

Cell migration of KFs was assessed using a transwell chamber. The upper compartment was added with serum-free medium comprising KFs (1 × 10^4^ cells/well), whereas 500 *μ*l of DMEM comprising 10% FBS was supplemented to the bottom compartment. After incubation, migrated cells were fixed and stained. The number of stained cells was counted under an inverted microscope (Olympus, Tokyo, Japan).

### 2.8. Immunofluorescence Staining

The subcellular localization of endogenous Smad proteins including smad2 and smad3 was determined using an immunofluorescence study as previously described [12, 13] using the same primary antibodies as used in the WB analysis and FITC-conjugated goat anti-rabbit second antibody (1 : 100; Abcam). Pictures were captured with a digital camera coupled with a fluorescent microscope (Olympus).

### 2.9. Statistical Analysis

All data are analysed via SPSS and represented as the mean ± SD. Student's *t*-test and one-way ANOVA were applied for the comparisons. *p* < 0.05 was considered as statistically significant.

## 3. Results

### 3.1. CTRP3 Expression in Keloid Tissues and KFs

As indicated in Figure 1(a), CTRP3 mRNA was markedly downregulated in keloid tissues compared with normal tissues. Consistently, downregulated protein levels of CTRP3 were also observed in keloid tissues (Figure 1(b)). In *in vitro* assays, the CTRP3 expression was lower in KFs than that in NFs at both mRNA and protein levels (Figures 1(c) and 1(d)).

### 3.2. CTRP3 Inhibited the KF Proliferation and Migration

To determine the function of CTRP3 in keloid, we applied pcDNA3.1-CTRP3 to overexpress CTRP3 in KFs. Results of WB proved that CTRP3 protein level was greatly induced by transfection with pcDNA3.1-CTRP3 in TGF-*β*1-treated KFs (Figure 2(a)). MTT assay showed that TGF-*β*1-induced KF cell proliferation was prevented by pcDNA3.1-CTRP3 (Figure 2(b)). In addition, the enhancement of KF migration caused by TGF-*β*1 was mitigated by pcDNA3.1-CTRP3 (Figure 2(c)).

### 3.3. si-CTRP3 Promoted the KF Proliferation and Migration

In Figure 3(a), the protein expression level of CTRP3 was observed to be dramatically reduced by si-CTRP3 in TGF-*β*1-treated KFs (Figure 3(a)). We found that downregulation of CTRP3 caused a significant enhancement of cell proliferation in TGF-*β*1-induced KFs (Figure 3(b)). Besides, knockdown of CTRP3 also promoted the migration of KFs under TGF-*β*1 induction (Figure 3(c)).

### 3.4. CTRP3 Inhibited the ECM Accumulation of KFs

Subsequently, as indicated by RT-qPCR analysis, TGF-*β*1-induced Col I, fibronectin, and *α*-SMA were markedly suppressed by CTRP3 overexpression (Figures 4(a)–4(c)). Besides, the Col I, fibronectin, and *α*-SMA protein levels were greatly upregulated in response to TGF-*β*1 stimulation, whereas they were inhibited by CTRP3 overexpression (Figure 4(d)).

### 3.5. si-CTRP3 Promoted the ECM Accumulation of KFs

The increase in Col I, fibronectin, and *α*-SMA mRNA induced by TGF-*β*1 in KFs was enhanced by si-CTRP3 (Figures 5(a)–5(c)). Furthermore, WB showed that the TGF-*β*1-induced protein levels of Col I, fibronectin, and *α*-SMA were greatly promoted by si-CTRP3 (Figure 5(d)).

### 3.6. CTRP3 Inhibited the TGF-*β* RI and TGF-*β* RII in KFs

TGF-*β*1 significantly induced the mRNA and protein levels of TGF-*β* RI and TGF-*β* RII in KFs. Nevertheless, apparent decreased levels of TGF-*β* RI and TGF-*β* RII were detected in CTRP3-overexpressing KFs (Figures 6(a) and 6(b)).

### 3.7. CTRP3 Regulated TGF-*β*/Smad in KFs

The nuclear translocation of smad2 and smad3 was determined using immunofluorescence staining. In Figures 7(a) and 7(b), TGF-*β*1 caused marked increases of smad2 and smad3 nuclear localization, which were attenuated by CTRP3 overexpression. In addition, the results of WB assay showed that TGF-*β*1 treatment obviously promoted the phosphorylation of smad2 and smad3 in KFs. However, the changed levels of p-smad2 and p-smad3 were mitigated by CTRP3 overexpression (Figure 7(c)).

## 4. Discussion

Keloid is related to excessive ECM protein accumulation, which are resulted from effusive production of cytokines and fibrogenic growth factors [14, 15]. A great deal of cells promotes the fibrosis process and contributes to keloid scarring. Among these cells, fibroblasts are thought to be central and responsible for the production of ECM-related proteins [14]. Compared to NKs, KFs are more sensitive to cytokines and fibrogenic growth factors. Additionally, the proliferation of KFs is increased, while apoptosis is reduced. These events further contribute to ECM deposition and fibrosis process.

Previous study proved that CTRP3 expression dysregulation has been found to be bound up with the severity of renal fibrosis. CTRP3 knockdown facilitates the TGF-*β*1-induced fibrotic changes in tubular epithelial cells, while CTRP3 overexpression attenuates fibrotic changes [16]. CTRP3 attenuates ECM production and myofibroblast differentiation, indicating that CTRP3 inhibits cardiac fibrosis [17]. CTRP3 is lowly expressed in liver fibrosis tissues and regulates the HSC propagation and migration, as well as ECM in response to TGF-*β*1 [18]. CTRP3 can inhibit TGF-*β*1-induced expression of smooth muscle agonist proteins and reduce the production of connective tissue growth factors and type I and type III collagen fibers; the local overexpression of CTRP3 in myocardial can inhibit myocardial interstitial fibrosis. These results indicate that CTRP3 has an antifibrotic effect in various tissues. We found that CTRP3 overexpression controlled TGF-*β*1-induced propagation, migration, and ECM accumulation in KFs, implying that CTRP3 promoted the fibrosis process in keloid scarring.

Cytokine TGF-*β*1 possesses broad biological functions, especially cellular differentiation and proliferation [19]. TGF-*β*1 is implicated in the processes in active wound healing, such as cell proliferation, inflammation, angiogenesis, ECM protein expression, and wound remodeling, which are mediated by Smad signaling [20]. Upon binding on TGF-*β*1, the dimerized TRIIs recruit and phosphorylate the TRIs, which phosphorylate the receptor-regulated smad2 and smad3 [21]. Subsequently, heterologous complexes of phosphorylated smads and smad4 are formed and then move to nucleus to regulate the target gene transcription, including Smad7 [21]. Smad7 regulates the TGF-*β*1/Smad pathway and prevents TGF-*β*1-mediated fibrosis [22, 23].

TGF-*β*1/Smad signaling functions a stimulator for wound repair and tissue regeneration in keloid pathogenesis [24–26]. TGF-*β*1 is currently known to be the most closely related to scar fibrosis of a cytokine. The Smad protein family is a TGF-*β* receptor downstream signaling protein discovered in recent years, which transmits the signal after TGF-*β* receptor activation from cytoplasm to the nucleus, acting on the corresponding target gene and thus playing a role. Inhibition of the TGF-*β*1/Smad pathway can inhibit keloid fibroblast proliferation, invasion, and angiogenesis and reduce collagen accumulation. Targeting TGF-*β*1/Smad signaling may be used for the prevention of keloid [27–30]. Cheng et al. [18] reported that CTRP3 attenuates the activation of HSCs through TGF-*β*/Smad signal path. Besides, CTRP3 was found to regulate Smad3 activation and thereby attenuate postinfarct cardiac fibrosis [17]. Our results showed that CTRP3 diminished the TGF-*β* RI and TGF-*β* RII in TGF-*β*1-induced KFs. Moreover, CTRP3 prevented the nuclear translocation of smad2 and smad3, suggesting that CTRP3 exerted its role via regulating TGF-*β*1/Smad [31]. It is the first study to explore the relation between keloid with CTRP3 with some limitations. In this study, only differences in expression between keloids and adjacent tissues were compared but not between normal skin tissue differences. In addition, the sample size of this study was also small, and the basic conditions of the included patients were not compared.

## 5. Conclusion

Within the inhabitation of TGF-*β*1/Smad, CTRP3 exerted an antifibrotic role in TGF-*β*1-induced KFs via inhibiting propagation, migration, and ECM accumulation. CTRP3 has the potential to be a new target for keloid treatment in the future.

## Figures and Tables

**Figure 1:** Quantification of CTRP3 expression in keloid tissues and KFs. The relative mRNA and protein levels of CTRP3 in keloid tissues and normal tissues were determined by RT-qPCR and WB (a, b). The relative mRNA levels of CTRP3/*β*-actin in KFs and NFs tested by RT-qPCR (c). The relative protein levels of CTRP3/*β*-actin in KFs and NFs tested by WB (d). ^∗^*p* < 0.05 vs. NFs.

**Figure 2:** Examination of cell proliferation and migration in CTRP3-overexpressing KFs. KFs were transfected with pcDNA3.1-CTRP3 or pcDNA3.1 to overexpress CTRP3. (a, b) RT-qPCR and WB were conducted to examine the mRNA and protein levels of CTRP3 after 48 h posttransfection in TGF-*β*1-stimulated KFs (a). MTT assay was conducted to assess cell proliferation (b). Transwell assay was performed to detect cell migration (c). ^∗^*p* < 0.05 vs. control KF group; ^#^*p* < 0.05 vs. TGF-*β*1+pcDNA3.1 group.

**Figure 3:** Examination of cell proliferation and migration in CTRP3-silencing KFs. KFs were transfected with si-CTRP3 or si-scramble to knock down CTRP3. RT-qPCR and WB were conducted to examine the mRNA and protein levels of CTRP3 after 48 h posttransfection in TGF-*β*1-stimulated KFs (a). MTT test was conducted to assess cell proliferation (b). Transwell test was performed to detect cell migration (c). ^∗^*p* < 0.05 vs. control KF group; ^#^*p* < 0.05 vs. TGF-*β*1+si-scramble group.

**Figure 4:** Examination of ECM accumulation in CTRP3-overexpressing KFs. The accumulation of ECM components including Col I, fibronectin, and *α*-SMA was examined by RT-qPCR and WB. Quantification of mRNA levels of Col I, fibronectin, and *α*-SMA (a–c). The protein expression levels of Col I, fibronectin, and *α*-SMA were tested via WB (d). ^∗^*p* < 0.05 vs. control KF group; ^#^*p* < 0.05 vs. TGF-*β*1+pcDNA3.1 group.

**Figure 5:** Examination of ECM accumulation in CTRP3-silencing KFs. The accumulation of ECM components including Col I, fibronectin, and *α*-SMA was examined by RT-qPCR and WB. Quantification of mRNA levels of Col I, fibronectin, and *α*-SMA (a–c). The protein expression levels of Col I, fibronectin, and *α*-SMA were tested via WB (d). ^∗^*p* < 0.05 vs. control KF group; ^#^*p* < 0.05 vs. TGF-*β*1+si-scramble group.

**Figure 6:** Examination of TGF-*β* RI and TGF-*β* RII expressions in CTRP3-overexpressing KFs. After transfection with pcDNA3.1-CTRP3 or pcDNA3.1 for 48 h, the mRNA and protein levels of TGF-*β* RI and TGF-*β* RII were detected via RT-qPCR (a) and WB (b). ^∗^*p* < 0.05 vs. control KF group; ^#^*p* < 0.05 vs. TGF-*β*1+pcDNA3.1 group.

**Figure 7:** Examination of the effect of CTRP3 on TGF-*β*/Smad signaling pathway. The subcellular localization of Smad2 and Smad3 was determined using immunofluorescence staining (a, b). WB was conducted to examine the levels of p-Smad2, Smad2, p-Smad3, and Smad3 (c). ^∗^*p* < 0.05 vs. control KF group; ^#^*p* < 0.05 vs. TGF-*β*1+pcDNA3.1 group.

## Data Availability

The datasets used during the present study are available from the corresponding author upon reasonable request.
